# A Statistical Synopsis of COVID-19 Components and Descriptive Analysis of Their Socio-Economic and Healthcare Aspects in Bangladesh Perspective

**DOI:** 10.1155/2023/9738094

**Published:** 2023-02-13

**Authors:** Mahtab Uddin, Kazi Shawpnil, Shafayat Bin Shabbir Mugdha, Ashek Ahmed

**Affiliations:** ^1^Institute of Natural Sciences, United International University, Dhaka 1212, Bangladesh; ^2^Department of Computer Science & Engineering, United International University, Dhaka 1212, Bangladesh

## Abstract

The aim of the work is to analyze the socio-economic and healthcare aspects that arise in the contemporary COVID-19 situation from Bangladesh perspective. We elaborately discuss the successive COVID-19 occurrences in Bangladesh with consequential information. The components associated with the COVID-19 commencement and treatment policy with corresponding features and their consequences are patently delineated. The effect of troublesome issues related to the treatment is detailed with supporting real-time data. We elucidate the applications of modern technologies advancement in epidemiological aspects and their existent compatibility in Bangladesh. We statistically analyze the real-time data through figurative and tabular approaches. Some relevant measures of central tendency and dispersion are utilized to explore the data structure and its observable specifications. For a clear manifestation, *Z*− scores of the COVID-19 components are analyzed through the Box-Whisker plot. We have discovered that the gathered data exhibit features that are unsatisfactory for the normal distribution, are highly positively skewed, and are predominated by the earliest occurrences. Infections and deaths were initially lower than the global average, but they drastically rose in the first quarter of 2021 and persisted for the remainder of the year. Substantial preventive results were produced by the region-wisetime-worthy moves. In the fourth quarter of 2021, the infections and deaths noticeably decreased, and the number of recoveries was highly significant. In the middle of 2022, a lethal rise in infections was observed in Bangladesh and that was quickly stabilized, and the pandemic ingredients were under control. According to our assessment, some concluding remarks are made at the end of this work.

## 1. Introduction

Epidemiology refers to the cogitation and exploration of the spreading and natural attributes and forecasting of the public health risk factors assessed for a demonstrated population [1]. It is essentially related to the studies of the demographic behaviors of any target community. Due to the requirement of preventive measures the contemporary public health-related issues with the emergence of the betterment of healthcare technologies, the term epidemiology is now getting significant attention with practical importance [2]. Epidemiology is compactly relevant to infectious diseases, such as HIV, AIDS, influenza, tuberculosis, Ebola, Nipah, and Zika [3].

Presently, highly contagious COVID-19 is the most conspicuous epidemiological phenomenon involving mysterious mechanisms of transfusions. In early 2020, after the December 2019 escapade at the city of Wuhan in China, the World Health Organization (WHO) proclaimed potentially severe acute respiratory syndrome coronavirus 2 (SARS-CoV-2) as the perpetrator of grievous COVID-19 [4]. This natural disaster rapidly expanded almost all corners of the globe, including Bangladesh.

COVID-19 has a detrimental influence on many elements of society and is especially harmful to individuals who belong to the most vulnerable social groups. The unimpeded natural world of nonhumans conceals humanity. According to WHO, outdoor air pollution kills 7 million people worldwide each year, and more than 80% of the civil population is exposed to polluted air. More than 4 million deaths each year are globally caused by heart illnesses, strokes, lung cancer, chronic lung diseases, and respiratory infections (https://www.who.int/health-topics/air-pollution). Those issues were affected much more during the COVID-19 pandemic. Air quality and climate play an important role in the COVID-19 situation. During the lockdown, it is noticed that most of the hospitals were in deadly condition due to the lack of a hygienic atmosphere.

SARS-CoV-2 is an RNA-based virus that is a frantically transmissible virus with volatile strains and epidemic variants over the world [5]. Consequently, some irregular and successive transmission waves occurred in recent times. The number and pattern of infections, deaths, and recoveries due to COVID-19 are varying with different variants [6]. Some variants of SARS-CoV-2 are eminently lethally and have no geographical bound. The horrific infectious genre of COVID-19 is now declared a pandemic by the WHO [7].

Bangladesh is a developing country in South Asia that is naturally beautiful. The economy of Bangladesh is progressing rapidly and is in the way to acquire the Sustainable Development Goals (SDGs). It is noticed that every sphere of life including women empowerment has immensely developed in the last decade. However, the outbreak of COVID-19 has affected every sector of Bangladesh intensely [8]. In Bangladesh, community transmissions started and climbed exponentially in the first quarter of 2020.

Earlier to the COVID-19 pandemic, the economy of Bangladesh was rising swiftly and earned on average a 7% increase in annual income. But due to the impact of the pandemic, according to the Bangladesh government, the rate of increase in annual income came down to 5.2%, whereas the government expected it to be 7.5% (https://www.unido.org/media/64590).

The pandemic COVID-19 has had a vital impact on the global economy. According to the International Monetary Fund (IMF), till now, the global economy is decreased by 4.9% due to COVID-19 which is higher than any other consequence. The safety measures against COVID-19 significantly reduced the workplace and workforces that remarkably hampered worldwide trade and business. The International Labor Organization (ILO) reports nearly 1.6 billion workers lost their livelihoods which is about 50% of the total labor. More than half of global employers in several business and economic sectors are suffering from the effect of COVID-19. The manufacturers, retail traders, and service-providing authorities are facing terrible hardship during COVID-19. As a part of the world economy, Bangladesh's economy was also severely invaded by the crisis of COVID-19. The readymade garments sector is drastically fallen due to inactivity from the importers. Medium and small business entrepreneurship is about to destroy and service-providing institutions sent off the majority of their workers because of no work due to the lockdown. People of lower or lower-middle income suffered the most as they had no deposits for future survival. Almost people in every economic class are downgraded within the contemporary COVID-19 pandemic, and the chain of socio-economic command structure is about to be badly impacted. Moreover, the agricultural sector of Bangladesh is damaged due to the transportation shortage during the lockdown. Detailed information about the world-wide economic crisis and compare to the situation in Bangladesh can be found in the Booklet published by the United Nations International Children's Emergency Fund (UNICEF) (https://www.unicef.org/bangladesh/media/5256/file).

The government of Bangladesh announced the outbreak of the COVID-19 virus in March 2020. The Institute of Epidemiology, Disease Control and Research (IEDCR), the epidemiology institute of Bangladesh reported the first three known cases on 8 March 2020 [9]. The virus was spreading gradually over the county from then, and the number of infected cases also increased. The Directorate General of Health Service (DGHS) announced daily reports; due to community transmission, 48 confirmed cases and 5 deaths are found on 28 March 2020 [10].

People who had any form of respiratory distemper are the vital sufferers of COVID-19. Even someone who recovered from COVID-19 infection experienced long-term lung complexity [11]. Elderly citizens and patients with chronic diseases, such as cardiovascular disorder, diabetes, and other respiratory illness, are mainly affected by COVID-19 spreading waves [12]. The COVID-19 virus can transmit from the infected people's mouths or noses as small liquid objects through cough, sneezing, and breathing with a range from aerosols to droplets.

Medical experts are worried about not having enough test kits to identify the infected people in the country. Newspaper, print media, and social media telecasted the latest news, awareness, and symptoms of COVID-19 [13]. The government opened isolation centers over the country. The COVID patient stayed in those isolation centers or home quarantine. During the pandemic, people of Bangladesh faced a shortage of medical-grade oxygen and intensive care unit (ICU) [14].

Though several vaccines are discovered and a remarkable number of people are vaccinated worldwide, due to the consecutive appearance of newer variants no absolute preventive steps are found to impede COVID-19. Some public awareness steps are taken globally to minimize the massive number of infections, such as quarantine, isolation, and lockdown [15]. There are many reasons behind the lack of success in COVID-19 treatment that governments of many countries initiated, namely, poor medical infrastructure, communication breaches and lack of authenticity of the gathered information, and ignorance and unwillingness to the treatment from the side of civil populations [16].

During the spreading of COVID-19, a large number of studies are ongoing worldwide. A detailed analysis of the COVID-19 situation in China is statistically portrayed in [17]. The significance of several parameters of COVID-19 infection in Saudi Arabia is statistically analyzed in [18]. A regression analysis-based prediction strategy for COVID-19 infections in India is studied in [19]. The statistical measures of the factors behind the community transmission of COVID-19 in Pakistan through real-time data are provided in [20]. A comparative analysis of COVID-19-related deaths in urban and rural arrears of the United States is discussed via statistical data illustrated in [21]. Recently, based on the comprehensive data of COVID-19 in Thailand, reconstructive transmission dynamics via stochastic modeling technique is studied in [22].

In this work, we are willing to elaborately discuss the socio-economic and healthcare scenario of COVID-19 spreading from the perspective of the people of Bangladesh, including the components of the treatment and accompanying troublesome issues that obstruct the treatment strategies. The discussion includes the impact of the age of information and the Internet of Things on the COVID-19 situation and their applicability in Bangladesh. The statistical manifestation and analogous discussions with recommending opinions will be provided as well.

## 2. Methodology

The present work can be partitioned into two basic categories. One is the descriptive analysis of the COVID-19 situation and associated socio-economic and healthcare aspects, and the rest is the statistical analysis of real-time data collected from various authentic sources.

In the beginning, the progression of COVID-19 in Bangladesh is narrated sequentially in Section 3. The commencement of COVID-19, sequential phenomena, and information about the healthcare authorities, and the monitoring body in Bangladesh are discussed in this section. Sections 4 and 5 consist of the components of COVID-19 and the issues impeding COVID-19 treatment in Bangladesh, respectively. The description of lockdown, quarantine, isolation, variants, and vaccinations are included in Section 4. In contrast, the reasons behind the impediment of COVID-19 treatment, such as ignorance and unwillingness of the mass people, scarcity of treatment facilities, the effect of different variants, economic crisis, and the impact of illiteracy are provided in Section 5.  Section 6 covers the discussion on the importance of the age of information and the Internet of Things in the safety measures for COVID-19. The situation of those factors in Bangladesh is included in this section as well.

Section 7 contains the main task of this work. The mechanism of collection and their statistical analysis are included in this section. Both graphical and tabular approaches are applied to manifest the real-time data of COVID-19 in Bangladesh. For an understandable analysis, measures of central tendency and dispersion are investigated along with an inquiry into *Z*-scores of the COVID-19-related components. Graphical and narrative analyses of every component are explored individually. Also, a detailed observation of the vaccination processes is delineated. Time, place, and the wave-based analysis of COVID-19 components are presented. The findings and discussion are made in Section 8.

## 3. COVID-19 Spread in Bangladesh

In this section, commencement of COVID-19 in Bangladesh, sequential phenomena, and the healthcare authorities along with the monitoring body are discussed.

### 3.1. Commencement of COVID-19

In Bangladesh, the very first confirmed case of COVID-19 was found on 3rd March 2020. On 18th March 2020, three nonresident Bangladeshi males returned from Italy and Kuwait along with a female, and the next day a family consisting three members returned from Italy once again. Those people had the symptoms of COVID-19 and that enhanced the community transmission of the COVID-19 [23]. The maiden death due to the outspread of COVID-19 was occurred on 21st March 2020. On 22nd March, a doctor died and many people found infected. Up to 23rd March 2020, in total, 23 healthcare workers were found to be infected; two more returnee were from India and Bahrain. Some returnee from Saudi Arabia and 4 locals were identified with COVID-19 morbidity on 24th March 2020; another death of the female that happened was linked to the community transmission [24]. On 3rd May 2020, recovery rates were grown up and reached to 1000 according to the governing authorities. On 13th June 2020, the total number of COVID-19 cases in Bangladesh exceeded the total number of COVID-19 cases in China. Just after two days of exceeding the total number of infections, the total number of recoveries from COVID-19 in Bangladesh has overtaken the total number of recoveries in China [25]. According to the government agencies of Bangladesh, up to 15th June 2020, about 15,000 patients were recovered from COVID-19. Many of the recovered people were not even recorded in the infected list, and outside the hospitals, many people recovered from COVID-19 infection by taking traditional home-made medications.

### 3.2. Sequential Phenomena

Initially, the people of Bangladesh were unaware of the deadliness of COVID-19 and hence apathetic to the healthcare rules and emergencies announced by the government. Due to the scarcity of skilled medical workers, a significant number of people were uncovered from the scheduled activities performed to handle COVID-19 spreading. As the consequence, community transmission happened rapidly [26]. Over time, the healthcare authority had taken the control of the situation and community transmission came to a submissive state. As Bangladesh is a densely populated country, the laboratories were insufficient for testing huge numbers of people. At the beginning, coronavirus cases were tested using only real-time reverse transcription-polymerase chain reaction (rRT-PCR) technique and, in December 2020, the government gradually increased the healthcare service facilities with hands-on training with the help of WHO [27]. To stop the prevalence of the virus, the government announced a “lockdown” throughout the country from 23rd March to 30th May and took some necessary steps to propagate the consciousness about the virus [28]. The country saw an elevated infection rate on 11th April 2020 which was the highest in Asia compared to March 2020. The government confirmed that all districts are under the cases on 6th May. The number of identified cases passed the number of identified cases in China, the country where the outbreak began by an unknown cause on 13th June. Moreover, Bangladesh reached the stern milestones of 160,000 cases and 2,000 deaths on 5th July. Some peaks were observed in the number of infections and deaths from July 2020 to June 2021, and then, both of them gradually came back to under hundred at the beginning of the year 2022 [29]. In contrast, the number of recoveries was trivial at the very first stage of the spreading of COVID-19 but it progressively grew with the initiative taken by the government, and after June 2021, it attained a swift pace of increment, which provides relief from the lethal threat.

### 3.3. Healthcare Authorities and the Monitoring Body

To superintend the COVID-19 situation and make crucial decisions, significance of the healthcare organizations and their monitoring bodies are unavoidable. The DGHS of Bangladesh is the principal authority to observe, analyze, and make decisions on public health issues, which remained invariant in COVID-19 affairs as well. DGHS collected, stored, and published the statistical data related to COVID-19 [30]. It also circulated public instruction and recommendations for the dues of the government in this pandemic situation. In parallel to the DGHS, mass people could collect the COVID-19 related information from Corona Info, which consisted of the figurative data representation related to COVID-19 in Bangladesh. IEDCR is an experimental research institute under government support that is functioning on infectious and epidemiological diseases in Bangladesh and their control. IEDCR worked in collaboration with DGHS to make the COVID-19 situation feasible [31]. IEDCR provided some hotline numbers, e-mail addresses, and a Facebook page for people to contact if they suspect COVID-19 infection or need more information. The Ministry of Health of Bangladesh is the monitoring body for healthcare matters in Bangladesh, which was managed to best fit the collaborative activities of DGHS and IEDCR in the COVID-19 breakout.

## 4. Components Related to COVID-19 Treatment

The immensely infectious COVID-19 outbreak affected all over the country's healthcare system and transmitted to mass people at an expeditious pace. COVID-19 is a new form of deadly virus SARS-CoV, which is transmissible between humans in diverse ways. In the beginning, the treatment procedure for this disease is poorly understood, and keeping social distance, wearing mask, and maintaining apt sanitation were the basic forms of treatment [32]. Then, some form of institutional activities for controlling COVID-19 is initiated, for instance, isolation, quarantine, and lockdown. Since COVID-19 is an RNA-based virus that is able to change its strain, there were several variants found, and still, new variants are coming in sequence. So, treatment of COVID-19 infection was obtrusive [33]. Time-demanding vaccines were discovered, and vaccination campaigns were carried out throughout the country later on. There were some vaccines discovered, commercially produced, and supplied by some worldwide renewed medicare companies supported by WHO. The conspicuous and prominent components related to the treatment of COVID-19 are discussed below.

### 4.1. Lockdown

Social distancing was one of the eminent options to reduce the community transmission of the COVID-19 infection. As the requirement of the treatment policy of COVID-19, the government of Bangladesh declared a zone-wise lockdown in the country several times [34]. In order to handle the COVID-19 crisis, the lockdown was retained by shutting down everything but hospitals and other healthcare facilities.

At airports, the authorities were watchful to detect any infection in passengers who were traveling from aboard (https://www.theindependentbd.com/post/233343). Travelers who had 100 degree Fahrenheit body temperature were examined through thermal cameras. Then, in Bangladesh, the first three confirmed cases reported positive as COVID-19 patients on March 8, 2020 (https://crisis24.garda.com/alerts/2020/03/bangladesh-first-cases-of-COVID-19-confirmed-march-8) and immediately shifted to hospital. One of them was announced first death from coronavirus by the healthcare officials on 18th March 2020 at Dhaka (https://www.reuters.com/article/health-coronavirus-bangladesh-idUSL4N2BB384) [30]. After that, on 22nd March, the government declared the first lockdown to reduce the spread of the COVID-19 and except emergency services all the public and private sectors were shut down (https://archive.dhakatribune.com/bangladesh/2020/03/23/govt-offices-to-remain-closed-till-april-4). In the meantime, the hospitals were preparing for the treatment procedure and laboratory experts for testing samples of the suspected patients who have coronavirus so that they can take necessary steps for the COVID-19 positive patients [35].

But the testing rate raised from mid-March, so the Bangladesh government again announced a second lockdown as the second wave arrived with an alarming turn in the country (https://archive.dhakatribune.com/bangladesh/2021/04/17/experts-bangladesh-s-second-COVID-wave-has-peaked-situation-likely-to-improve-in-may). Meanwhile, it was reported that with the prolonged lockdown, the academic activities immensely fell down and educational institutions went under severe uncertainties [36].

Bangladesh regularly rose up to new cases and the third wave with a new variant came up in a disaster situation. So, another lockdown was declared by the government, and the Bangladesh Army (BA) and Border Guard Bangladesh (BGB) deployed to stop people leaving their house without any emergency (https://archive.dhakatribune.com/bangladesh/2021/06/25/bangladesh-goes-into-nationwide-hard-lockdown-from-june-28). But for the sake of livelihood and the mild rate of the virus spread, the lockdown period ends [37].

Minimum 32 Bangladeshi people died of COVID-19 in the first week of July 2022. As a result, Bangladesh government declared a campaign, named “no mask, no service” in all official and public locations. Thus, an implicit lockdown imposed due to this sudden raise of the death rate (https://www.aljazeera.com/news/2022/7/6/fourth-wave-dozens-die-of-covid-in-last-5-days-in-bangladesh). Detailed information about the waves is unveiled in Table 1, and lockdown of COVID-19 in Bangladesh is unveiled in Table 2. It is to be noted that no salient lockdown is imposed in the fourth wave of COVID-19 in Bangladesh.

### 4.2. Quarantine

The term quarantine refers to keeping people away from the social interaction. During the pandemic like COVID-19, due to the chain of lockdown, there was no choice for the people and they had to quarantine themselves. When COVID-19 started in Bangladesh, due to financial and social phenomena, people had to work together and many of them were silent carriers of COVID-19. As a result, many of the workers and labors had to go under quarantine [38]. Many healthy people were finding it difficult to survive in such a condition, and everyone had to observe quarantine for few days. After completing the quarantine period, some of the suspected incoherent people quarantined themselves for at least two weeks apart from others as they found mild symptoms of COVID-19. In contrast, others went back to the society due to no further symptoms of COVID-19.

There are some protocols imposed by the government during the quarantine for controlling COVID-19 in Bangladesh. Measures are taken to increase social distancing among the people to limit or stop the transmission of the virus. This includes avoiding large gatherings, limiting the number of visitors to your home, working from home, maintaining safe distances from others, contacting friends and family online rather than in person, and if necessary, wearing personal protective equipment (PPE) [39]. As a result, the spread of the virus has slowed down reducing the maximum number of patients, thereby easing the strain on hospital infrastructure and needs. Because of quarantine, the maximum number of cases caused by the virus eases the pressure on resources and hospital demand is reduced by slowing the spread of the virus.

Physical activity decreased, lack of social interaction, and staying home is a boredom; these caused problems among people. Restriction of social interaction and not going out made things way beyond complicated at a stage of pandemic. The fear and anxiety level increased within the people, and working from home was not easy for all. In Bangladesh, the study of psychological behavior within quarantine is mainly affiliated with stress and loneliness symptoms [40].

A study on the quarantine in Bangladesh perspective portrayed that the effects of the home quarantine is profoundly connected to the psychological aspects and had noteworthy impact on psychological matters throughout COVID-19 pandemic. Lack of healthcare awareness, medical opportunities, and monetary assurance were the most noticeable impediments of the quarantine process in Bangladesh [41].

### 4.3. Isolation

The word “isolation” originates from the fact that the incidence of COVID-19 is increasing and people are not being given any place in the hospital. In such a situation, doctors advised that it would be wise not to come to the hospital unless the condition is very critical now. Before going into isolation, they were divided into two categories and the two types of people were kept in isolation: those who have been tested for COVID-19 and those who have not. Some of the isolated people had lack of oxygen saturation and were treated as infected and were needed to take medicare. Later, some people recovered and some of them died [42]. It was found that the number of recovered patients was increasing day by day and reduced the rate of affected patients after the isolation.

Some people took isolation in a negative way. During the sickness due to the COVID-19 infection, in the isolation period surviving alone seemed to be very tough and it greatly affected the people psychologically. Anxiety and fear of death came across their minds in that dangerous time of COVID-19. Some diseases stayed forever with them after suffering from COVID-19. So, this is a concerning topic to discuss otherwise they cannot fight with the virus [43]. Our body reacts how we want it to react, so if anxiety and depression grab you, then it would be very difficult to turn back. Isolation is marked as one of the prominent catalysts of mental instability during COVID-19.

In Bangladesh, some people researched it, and according to their analysis, it is observed that more than 50% isolated people suffered from anxiety and depression; to be exact, they are 52.7% and 52.2%, respectively. Out of them, a significant number of isolated people had acute manifestation of anxiety and depression, which is definitely a fatal extent [44]. Dealing with the pandemic situation was not easy for everyone to handle alone. Every family does not have separate rooms for all the members; during that time, if one member is COVID-19 positive, it is very difficult to manage and keep everyone safe. Also, those who were isolated cannot be taken care of by others. Some cases with suicidal attempt were also noticed throughout the pandemic period [45]. A meta-analysis exhibited that pervasiveness of anxiety and depression among the isolated people with COVID-19 is remarkable and statistically their rates are 47% and 45%, respectively [46].

### 4.4. Variants

As the virus spreads, new variants or versions of the virus can appear. Variations usually do not affect the function of the virus. But sometimes, they change their behavior. Researchers worldwide are surveying the differences in the virus that cause COVID-19 (https://www.jagranjosh.com/general-knowledge/variants-of-sars-cov-2-in-the-world-covid-19-variants-1623846555-1). Contemporary research is helping scientists to better understand how COVID-19 mutations might affect human health if some spread faster than the others [47].

The entire genetic structure of the coronavirus is contained in RNA (ribonucleic acid). Though not identical, RNA and DNA have some similarities. When a virus infects a person, it binds to human cells, enters them, and makes copies of its RNA to help spreading. RNA is varied if a replication error occurs. Usually, viruses change their genetic structure and gain the transmission potential as they circulate among people over time [48].

We talk about “variants” when these modifications are entirely divergent from their original form. Scientists analyze the virus's genetic makeup to find variations and then check for differences to see if there are any changes. Variants of the SARS-CoV-2 virus, which produce COVID-19, have emerged and been detected in several countries worldwide following the global spread of the virus [49].

Another example is delta variant. WHO classified the delta version as a variant of concern on May 11, 2021, and it is currently the most widely circulated variant worldwide [50]. Compared to previous virus strains, the delta variant spreads faster and is responsible for more number of cases and deaths worldwide. The delta variant is protected against all licensed COVID-19 vaccines currently in use, and all of them are safe and effective [51].

It is perceived that in the third wave, when the delta variant was spreading, new cases rate rose up to 13,817 just before the lambda variant came up. Also, the highest number of deaths of 264 was found at that time.

Different variants came up with different symptoms which effected the treatment category for dealing with concerning cases. This became a directing factor in the treatment facility as well as in the general people for maintaining more safety. During lockdown, in different waves variety of variants took place in our country from the origins of the variants [52]. The variants of COVID-19 have diversified attributes. Some are highly infectious, some are very deadly, and some of them are ancestors of further healthcare complexities, especially, heart, kidney, and lung infections. So, the continuous arrivals of the variants of COVID-19 made the impediments of exact treatment approach, which enhanced the scarcity of the control of COVID-19 situation in Bangladesh [53]. In Table 3, the variants of COVID-19 detected in Bangladesh are delineated along with their origins and dates of detection.

### 4.5. Vaccinations

Vaccination is a primordial and prominent apparatus for preventing the infectious disease like COVID-19. To combat against COVID-19, vaccination is a safe zone for people because vaccine builds natural immunity to a disease in our body before we get sick or infected with some virus. On June 21, 2020, Bangladesh got the rights to proceed from China to vaccinate general people to fight with the lethal virus COVID-19 (https://archive.dhakatribune.com/health/coronavirus/2020/06/21/COVID-19-bangladesh-to-get-priority-if-china-develops-vaccine). It started from January 27, 2021, and Bangladesh government decided to start mass vaccination from February 07, 2021 with the Oxford-AstraZeneca vaccine (https://www.aljazeera.com/news/2021/1/28/bangladesh-starts-COVID-vaccination-drive) and targeted to reach 6 million doses in the first month and 5 more million within the next month (https://www.thedailystar.net/frontpage/news/historic-day-2035021). The COVID-19 vaccines which have been approved for use by WHO and assumed to be applied in Bangladesh are addressed below with a brief idea for each of them.

- AstraZeneca (Covishield) is a type of viral vector vaccine, originated from United Kingdom and developed by Oxford University and British-Swedish company, AstraZeneca. The vaccine is 81% effective against the alpha variant, and 61% against the delta variant [54].
- Sputnik V (Gam-COVID-Vac) is a type of viral vector vaccine, originated from Russia and developed by Gamaleya Research Institute of Epidemiology and Microbiology. Sputnik V produced antibodies capable of neutralizing the gamma variant [55].
- Sinopharm (BBIBP-CorV) is a vaccine of inactivated virus, originated from China and developed by Sinopharm's Beijing Institute of Biological Products. Initially, Sinopharm was found 86%effective (https://gulfnews.com/uae/health/uae-ministry-of-health-announces-86-per-cent-vaccine-efficacy-1.1607490555571). The effectiveness of Sinopharm against symptomatic cases was 78.1%, whereas it is found 100% effective for the severe cases [56].
- Pfizer–BioNTech (BNT162b2) is mRNA-based vaccine, originated from Germany and developed by the German biotechnology company BioNTech. American company Pfizer incorporated to BioNTech for the clinical trials, logistics support, and production of Pfizer–BioNTech vaccine in the process of development. Pfizer–BioNTech is 93.7% and 88.0% effective against alpha and delta variants, respectively [57]. Another version of Pfizer vaccine is called Pfizer-PF, which is initially introduced as an oral/nasal dose of vaccine effective for individuals of 12 years age and older [58].
- Sinovac (CoronaVac) is a vaccine made of inactivated virus, originated from China and developed by Chinese company Sinovac Biotech. Sinovac provided protective levels of measured antibodies against the omicron variant and found effective for the elderly patients against the gamma variant [59, 60].
- Janssen (Jcovden) is a type of viral vector vaccine, originated from Netherlands and developed by the collaboration with Belgian parent company Janssen Pharmaceuticals, a part of American company Johnson & Johnson. The Janssen vaccine can be applied for a person who is not fit to receive mRNA-based vaccines [61].
- Moderna (mRNA 1273) is an mRNA-based vaccine, originated from America and developed by American company Moderna, supported by the United States National Institute of Allergy and Infectious Diseases (NIAID) and the Biomedical Advanced Research and Development Authority (BARDA). Moderna is found to be effective for the delta variant [62]. Moderna is eligible for the treatment of pregnant women as well [63].

A viral vector vaccine produced through the genetic material coding for a target antigen within the recipient's host cells. An inactivated vaccine contains some virus, bacteria, or other cultivated pathogens and killed them for destroying the infectious viruses. An mRNA vaccine includes the messenger RNA (mRNA) to generate the internal immunity.

## 5. Troublesome Issues Accompanying to COVID-19 Treatment in Bangladesh

In this section, we will narrate some incommodious issues that engendered obstruction of COVID-19 treatment in Bangladesh. Some of them originated from the side of mass people due to illiteracy and passiveness, and the rest of them sprouted from the deficiency of systematic healthcare infrastructure and economic expediency.

### 5.1. Ignorance and Unwillingness to the Treatment

Most Bangladeshi people are not acquainted with the signs and impacts of pandemics. They were confused with the symptoms of COVID-19 and the other flu-related fevers. They had no idea about the aftershock of the waves of COVID-19 variants and were not aware of the lethality of this infectious disease. Due to the ignorance of the spreading of COVID-19 and unwillingness to the healthcare strategies, the community transmissions were elevated significantly [64]. Some of the people were naturally resistant to the infection owing to the presence of desired antibodies; this fact highly encouraged the uneducated and troublesome to be reluctant to the steps taken by the government to minimize the rate of COVID-19 infections. Some people were unnecessarily overconfident about their health issues and thought they will not be affected by the COVID-19 infections, which was another cause of unwillingness [65]. A few cases of ignorance were caused due to the deficit of trust in the COVID-19 protective measures. Overall paucity of proper healthcare education and insufficient knowledge about the pandemics are the fundamental source of ignorance and it made the Bangladeshi people unwillingness to the COVID-19 treatment, and hence, the rate of infection climbed conspicuously [66].

### 5.2. Lack of Treatment Opportunities

As a third-world country, Bangladeshi people face a lack of treatment opportunities due to insufficient infrastructure and scarcity of skilled healthcare personnel. During the COVID-19 period, the hospital conditions started worsening. It goes the same for those who admitted and those who could not get a single place in the hospital. Even some doctors did not attend the hospitals regularly at that time. Family members had to go through a tough time managing everything. Although the quality of medical equipment and standard training process are improving over time but they are yet to be plentiful for the extant demand [67]. The deficiency of the proper ventilation system and exiguous medication made the contemporary pandemic scenario awful. The people of Bangladesh are not habitual to infectious diseases like COVID-19; that is why the preparation to deal with COVID-19 was incommensurate [68]. Although much medical equipment was managed in the peak of the infection, the apathy of some of the healthcare authorities is another cause for the increment in the number of COVID-19 patients present in Bangladesh [69].

### 5.3. Break-Outs of Different Variants

The whole COVID-19 situation passes some difficult waves. Various types of variants came and went, but every variant came with new types of cases and symptoms. For every variant, the symptoms change with a new way of treatment pattern [70, 71]. COVID-19 treatment patterns need proper instructions before giving them to people. People with other illnesses should be concerned about the treatment procedure. But the lack of positivity and awareness people is making it difficult to get rid of it. This is a severe issue that needs to be solved among general people. Because it can break the infrastructure, it makes it difficult to modify if any new variants with new symptoms come [72].

### 5.4. Lower Economical Structures

Bangladesh is a developing country, and people who are under privilege do not maintain a healthy lifestyle. Poverty is the problem here; they cannot afford the cleaning products to maintain the COVID-19 precaution situation. Some of their lower-income occupations or lower economical ability do not support extra expenses [73]. People who drive rickshaws, laborers, and local shopkeepers cannot survive with the high precautionary system of COVID-19 [74]. Usually, they do not maintain a proper hygiene environment. For that, the awareness of hygiene is not proper enough for covering this situation. The first condition of COVID-19 is to maintain hygiene properly. But they do not have proper guidelines and a lack of awareness causes more suffering.

### 5.5. Superstitions and Rumors

Some people in society think that this whole pandemic situation and COVID-19 cannot do any harm to them. These superstitious things mislead some people from the real situation of COVID-19. So-called religious matters are sensitive cases but some people use them inappropriately and outspread wrong information. They think the almighty will save them without any medication; this pandemic is given for some reasons. This kind of illiteracy is leading people from ignoring the COVID-19 situation [75]. There was a rumor propagated that COVID-19 is an infectious disease in wintry countries and will not spread to warm countries like Bangladesh. As a consequence, people were leading their regular life without preventive measures which caused a higher rate of infection of COVID-19.

## 6. Impact of Age of Information and Internet of Things in COVID-19 Situation

In this section, we will discuss the importance and aptness of age of information and Internet of Things and their influence in epidemiological circumstances. Also, the present scenario of age of information and Internet of Things are highlighted according to Bangladesh.

### 6.1. Age of Information

The modernization of information is a burning issue in the present era of information technology because of its practical functionality [76]. A naturalistic data update process is significantly demanding, which consists of the composition of network-based data monitoring, tactical connections, multiconnecting modules, internet-based data station, human-computer interfaces, and physical security systems [77]. Due to lack of effectiveness and data modernity, classical communication devices are being replaced with updated and optimized data analysis tools [78]. AoI is an auspicious and potential assessment of data expediency that clarifies the adaptability and sustainability of the latest installed devices. For controlling the collaborative information updates with adequate credibility, the worth of AoI is unavoidable.

In the emergence of open-source feasibility and computer-aided data analysis, AoI has a crucial role. AoI is indispensable for the trustworthiness of collected data and their further accomplishment [79]. Statistical measures of the collected data must be highly contingent on their practical eligibility and aspects of biophysics, which are the preeminent features of AoI [80]. Assumption of the future circumstances according to the contemporary ambiance is obligatory, which can be empirically ascertained through the AoI [81]. In epidemiological situations, healthcare techniques can be contemplated according to the structure of the collected data, their accuracy, change of atmosphere over time, and the infrastructural ability of the healthcare authority [82, 83]. In those attributes, regularity and positiveness of the collected data are the most important aspects, which can be justified through AoI [84]. AoI is tightly connected with the methodological updates and enhancement of their systematic utilization for statistical analysis of epidemiological factors [85]. In the existent COVID-19 pandemic, optimal accuracy of the collected data is inescapable due to the safety measures and decision-making for treatment strategies, which is linked to AoI rigorously [86].

### 6.2. Internet of Things

In the present day, the Internet of Things (IoT) is playing a key role in the advanced technologies of the data collection process and their statistical analysis [87]. Assignation of IoT is exigent for the convenience of storing allotment in computing devices, efficient data dissemination, and rapid access to remote data servers [88]. Recently, Artificial Intelligence (AI) has been commonly incorporated with IoT, which can efficiently accumulate and categorize real-world data through remote sensors and their computational applications without the physical presence or human-based schemes [89, 90]. The term machine learning (ML) is deeply compacted to IoT for the purpose of statistical experiments, including similarity analysis, data forecasting, and pattern recognition of real-time data with the optimal time and cost [91, 92]. In the current epidemiological calamity, the requirement of IoT is unavoidable due to the expeditious remote access to treatment-related information, distant workload distributions, and methodical updates from the decision-making healthcare officials [93].

ML processes for statistical modeling are becoming more standard in the literature of epidemiological studies. These techniques have the potential to vastly expand our understanding of health and the available interventions, far exceeding our existing capabilities [94]. To improve treatment outcomes, hospitals and research facilities will utilize AI to train machines to handle data rapidly and effectively. The functions that programs may carry out include treating strokes, identifying heart problems, and improving diagnostic radiology skills [95]. Being updated about the pertinent situation is essential for setting up the preventive measures against the community transmission and related components of COVID-19, which is the prime concern of IoT [96].

COVID-19 has caused immense suffering, loss of life, and death. The ease with which this form of coronavirus can spread highlights the flaws in many healthcare systems around the world. Many governments, scientific, commercial, and other institutions and interest groups around the world have fought the disease in various ways since its outbreak. Science and technology have helped several countries mitigate the effects of the pandemic and implement programs aimed at identifying and treating diseases. Modern technological methods, especially AI tools, are also being researched to track coronavirus transmission, identify those at a high risk of dying, and diagnose patients with the condition [97]. Detection and diagnosis of COVID-19 are essential to campaigns against the virus. Current noninvasive diagnostic analytical techniques include breast CT and chest X-ray imaging, bimolecular, serological, and viral throat swab tests [98]. Rapid and early diagnosis and surveillance of infected individuals are critical to contain epidemics and isolating viruses, and there is a desire for innovation in this area [99].

### 6.3. Scenario in Bangladesh

In Bangladesh, because of the factors mentioned in the previous section, preserving the fundamental features of AoI was immensely challenging and inconceivable for some affairs. Consequently, policymakers were in a dilemma at the initial stage of the COVID-19 situation. Gradually, the environment went under control at the beginning of 2021, and healthcare activities are feasible.

From Bangladesh's perspective, due to technological deficiency and insufficiency of skilled computer-based medical analysts, IoT is still not in the fully efficacious stage. But the situation compelled the advancement of IoT in Bangladesh during the existent epidemiological catastrophe. After the initial wave of COVID-19, the Bangladesh government took necessary steps to ensure the unbounded flow of information. Ministry of Health directly monitored the COVID-19 phenomena and maintained a public database, both on the website and regular announcements through various sources of social and printed media. Data analysts and medical professionals worked together for a smooth information flow under the guidance of government-affiliated healthcare institutions, namely, IEDCR and DGHS of Bangladesh.

## 7. Accumulation of Statistical Data of COVID-19 Components and Their Interpretative Analysis

In this section, statistical analysis of some COVID-19 occurrences in Bangladesh is portrayed through figurative and expository approaches. Prior to doing the statistical analysis the scheme of data collection referencing the appropriate sources and time period is stated elaborately. Measures of central tendency and dispersion are depicted for the real data and a more refined view is presented through *Z*− scores (standardized value) of COVID-19 components. We are aiming to discuss the number of tests, infections, deaths, recoveries, quarantines, isolation, and a detailed review of vaccinations.

### 7.1. Data Collection Scheme

We are working with a large amount of data having multiple ingredients, which needs a very reliable data sources but due to fragile infrastructure and proper guidelines, a single data source cannot fulfill the entire requisite information. So, we have collected and structured our aimed data-set from various national and international organizations, for instance, DGHS Bangladesh, (http://dashboard.dghs.gov.bd/webportal/pages/COVID19.php) Corona Info (https://corona.gov.bd), IEDCR, (https://iedcr.gov.bd/COVID-19/COVID-19-general-information), Worldometer (https://www.worldometers.info/coronavirus/country/bangladesh), WHO (https://www.who.int/emergencies/diseases/novel-coronavirus-2019/situation-reports), UNICEF Bangladesh (https://www.unicef.org/bangladesh/en/coronavirus-disease-COVID-19-information-centre), and Wikipedia (https://en.wikipedia.org/wiki/Statistics_of_the_COVID-19_pandemic_in_Bangladesh). We have gathered some informative data from local newspapers, social media, and news bulletins as well.

Here, we aimed to analyze the data up to 30th September 2022. For the number of tests, infections, deaths, and recoveries from 8th March 2020, whereas for number of quarantines and isolations the data are admissible from 20th December 2020. The data for vaccinations are available from 27th January 2021 for the first dose, 8th April 2021 for the second dose, and 21st December 2021 for the third dose.

### 7.2. Statistical Analysis

Measures of central tendency and dispersion of the components of COVID-19 in Bangladesh are included in this section. We consider the maximum daily cases, their average, quarterly positions as the measures of central tendency. On the other hand, mean deviation, standard deviation, and their coefficients (in percentage) are taken as the measures of dispersion.  Figure 1 demonstrates the abovementioned statistical measures of components of COVID-19 in Bangladesh.

The maximums of the COVID-19 components are far ahead of their average values. In comparison to the average values, the mean deviation and standard deviation are found very high. For almost every component, the mean deviation is about 100% of the average, whereas it is about 150% for the Standard deviation. Those measures of dispersion are close to 60% only for the number of tests. The measures of the quartiles display the nonequidistant positioning that indicates a nonuniform distribution of the target data. So, from the graphical testimony, it can be claimed that the COVID-19-related data are moderately scattered and have noticeable irregularity.

Since the magnitudes of the data of COVID-19 components are unequal, a collective comparison is not possible in their current values. As the remedy of this problem, the *Z*− scores of the desired components are estimated and exhibited them through a Box-Whisker plot as shown in Figure 2.

From the Box-Whisker plot, it is evident that distributions for all of the COVID-19-related components failed to maintain the characteristics of Normal distribution and skewed positively. The very long right tails of the distributions reveal that the averages of the components are greater than the modes but less than the medians. Thus, it is obvious that all of the components were very high initially and gradually diminished over time with some inconsistency.

### 7.3. Number of Tests

We are willing to investigate the daily number of tests (suspected cases) and the division-wise total number of tests in Bangladesh.

Figure 3 displays the daily number of tests from 8th March 2020 to 30th September 2022. There are some peaks indicating the extensive number of tests were done. The test includes polymerase chain reaction test (PCRT) and rapid antigen test (RAT). Three massive peaks are found on 12th April 2021, 3rd August 2021, and 25th January 2022 for number of tests 34,968, 55,284, and 49,492, respectively.

Figure 4 reveals the division-wise total number of tests in Bangladesh. From Figure 4, it is evident that highest number of tests occurred in the Dhaka division with 5,951,657 cases followed by the Chittagong division with 3,044,602 cases, whereas lowest number of tests occurred in the Barisal division with 311,092 cases.

### 7.4. Number of Infections

We investigated the daily number of infections (confirmed cases) and the division-wise total number of infections in Bangladesh.

Figure 5 displays the daily number of infections from 8th March 2020 to 30th September 2022. Some peaks are found indicating that a large number of infections happened. The noticeable peaks were on 7th April 2021, 28th July 2021, and 25th January 2022 for number of infections 7626, 16,230, and 16,033, respectively.

Figure 6 reveals the division-wise total number of infections in Bangladesh. From Figure 6, it is apparent that the highest number of infections occurred in the Dhaka division with 950,132 cases followed by the Chittagong division with 308,537 cases, whereas the lowest number of infections occurred in the Mymensingh division with 40,690 cases.

### 7.5. Number of Deaths and Recoveries

Figures 7 and 8 exhibit the countrywide daily number of deaths and recoveries in Bangladesh from 8th March 2020 to 30th September 2022.

Figure 7 depicts that the maximum number of deaths was observed on 5th and 10th August of 2021 with 264 deaths. Also, 112 deaths were occurred on 19th April 2021.

Figure 8 expounded that the topmost number of recoveries was attained on 8th August 2021 with 16,627 recoveries followed by 13,853 recoveries on 13th February 2022. Also, 7266 recoveries were viewed on 28th April 2021. A strange incident was observed on 15th June 2020 that number of recoveries abruptly lifted to 15,297, which is an irregular phenomenon. It might have happened due to some late entry of recoveries at a time.

### 7.6. Number of Quarantines and Isolations

The daily number of quarantines and isolations from 20th December 2020 to 30th September 2022 are exposed in Figures 9 and 10, respectively.

From Figure 9, it is obvious that the greatest number of quarantines were 10,333 on 30th July 2021. Another two discernible peaks are found for 3413 and 6037 quarantine cases on 22nd April 2021 and 26th January 2022, respectively.

From Figure 10, it is decisive that the largest number of isolations is 5138 on 27th July 2021 followed by 5022 isolations on 2nd August 2021. One more peak for isolations was found on 28th January 2022 with 2626 isolation cases.

### 7.7. Number of Vaccinations

The vaccination in Bangladesh was started on 21th January 2021. Initially, the AstraZeneca vaccine was introduced as the first dose of the vaccination. Second dose of the vaccination was started on 8th April 2021 with the AstraZeneca vaccine once again. The third dose (boaster dose) was started on 21st December 2021 with Pfizer vaccine. Six types of vaccines were used in Bangladesh. Up to 30th September 2022, in total, 303,634,312 vaccines were provided. Among the vaccine takers, numbers of male, female, and transgender were 151,062,898, 152,570,806, and 608, respectively. Sinopharm vaccine had the dominant role in total number of vaccinations for first and second doses, whereas Pfizer took the prime position in the total number of third dose of vaccinations. A brief idea of the vaccinations in Bangladesh is given in Table 4.

Figure 11 displays the number of daily vaccinations from 21th January 2021 to 30th September 2022, whereas Figure 12 shows the daily vaccinations for particular doses in the same time schedule.

Figure 11 represents that highest number of vaccinations were occurred on 26th February 2022 with 11,654,878 vaccinations, where first dose vaccinations were dominant with 10,603,093 cases. Two more noticeable days were observed on 28th March 2022 and 19th July 2022 with 7,282,537 (including 6523021 second dose vaccinations) and 5,911,842 (including 5637003 third dose vaccinations) vaccinations, respectively.

Figure 12 conveys the scenario of dose-wise vaccinations in Bangladesh. Up to 30th September 2022, in total, 131,600,634, 122,539,180, and 49,494,498 number of vaccines are distributed as the first, second, and third doses of vaccinations, respectively. The maximum number of first dose vaccines were distributed on 26th February 2022 accompanying 10,603,093 vaccines, which are 6,523,021 and 5,637,003 for second and third doses on 28th March 2022 and 19th July 2022, respectively.

The subfigures of Figure 13 illustrate the synopsis of the type-wise vaccinations with appropriate dates in Bangladesh for the first, second, and third doses, respectively, within the target time period. From Figures 13(a)–13(c), it is palpable that Sinopharm vaccine was the most widely distributed vaccine for the first and second doses, whereas Pfizer vaccine was major in the third dose of vaccination. On the basis of daily vaccinations, Sinovac, Sinopharm, and Pfizer vaccines were leading in the first, second, and third doses of the vaccinations, respectively. A comprehensive outline of type-wise maximum vaccinations including the dates is demonstrated in Table 5.

Note that, the vaccine Pfizer-PF was involved in the first dose of the vaccinations, whereas no Janssen vaccine was included in that dose.

Figure 14 portraits the division-wise vaccinations status in Bangladesh, whereas Table 6 conveys the summary of the division-wise vaccinations information.

Figure 15 discloses the district-wise vaccinations status in Bangladesh, whereas Table 7 apprises the summary of the district-wise vaccinations information. The vaccination coverage more than 100% indicates the number of vaccination exceeds the number of residences due to entry of people from other districts.

### 7.8. Wave-Wise Distribution of COVID-19 Components

Here, the wave-wise summary of the occurrences of the COVID-19-related components in Bangladesh is provided in tabular form.  Table 8 exemplifies the wave-wise distributions of the COVID-19 pandemic-related components at a glance.

## 8. Findings and Discussion

Statistical analysis of the data gathered from COVID-19 components conveys their nonuniform shape and irregular arrangement. The target data failed to acquire the pattern of Normal distribution with conspicuous positive skewness. For Bangladesh, the dominance of the causation of the components is observed at the beginning of COVID-19.

From the figurative comparisons of number of tests, infections, deaths, and recoveries, it is obvious that from the beginning to the third quarter of 2021 the COVID-19 situation in Bangladesh was very similar for all of the mentioned components. They had some noticeable cusps on July 2020, April 2021, August 2021, and January 2022, while the third one was the topmost. After January 2022, all of the mentioned components were gone down except some slight scatterings in July 2022. The number of tests, deaths, and recoveries are precisely followed the trend of the number of infections. The number of deaths was contemptible in comparison to the number of infections and clearly outplayed by the number of recoveries. In division-wise investigation, it was found that for both number of tests and infections, Dhaka division was at the pinnacle chased by the Chittagong division. But Barisal and Maymensingh divisions were at the undermost in the number of tests and infections, respectively. The number of quarantines and isolations defined the identical trend of the abovementioned components but data were mission before December 2020. They had unerringly the same aptitude of the number of infections in the timeline of their data availability. The number of quarantines was triumphed over the number of isolations, which is the indicator of the insufficiency of institutional amenities.

From the compendium of the type-wise vaccinations in Bangladesh for the doses, it is apparent that for the first and second doses Sinopharm vaccine was the dominant one, but Sinovac and Sinopharm vaccines were provided as daily maximum vaccinations in the first dose and second doses, respectively. Pfizer was the leading vaccine type in the third dose of vaccination and maximum daily vaccinations were recorded for the Pfizer vaccine as well. From the given diagram of division-wise vaccinations, it is distinctive that the Dhaka division was under the maximum coverage and the Barisal division was under the minimum coverage for both the first and second doses, while in the third dose of vaccinations the Khulna division advanced to the first position and the Mymensingh division went to the bottom with the coverage. From the District-wise vaccination coverage, it is identifiable that for the first and second doses of vaccination the Gazipur positioned maximum, whereas Chuadangla reached to the top for the third dose. The Jhalokati, Shariatpur, and Gaibandha settled to the bottom of the vaccination coverage for the successive doses.

From the wave-based distribution of the COVID-19 related components, it is intelligible that the third wave of the COVID-19 propagation was the most momentous for all of the components.

During the COVID-19 pandemic, every family in Bangladesh had a tough time managing their livelihoods and medical necessities. However, with the advancement of medical science, scientists discovered some effective vaccines that resulted comprehensively and helped the people to get back to our habitual life. In this case, if people were aware about some precautions from the beginning, they might be able to minimize the deadly losses. For example, they were alert enough in immigration so that without the affirmation no one was allowed to enter from foreign countries. By closing down transportation through the border, we could stop those COVID-19-infected peoples who entered. Also, following the lockdown strictly and correctly from the very beginning community transmission could be diminished. If we could maintain these steps, it might lessen the loss during the COVID-19 period.

## 9. Conclusion

In this work, we have discussed the COVID-19 spreading in Bangladesh including the initial situation with the sequential phenomena and authorities concerning the healthcare administration during the pandemic. The basic components related to the COVID-19 treatment and corresponding obligations are pointed out regarding circumstances in Bangladesh. We investigated the troublesome issues that impede the COVID-19 methodical treatment opportunities in Bangladesh. The socio-economic and healthcare issues are assimilated in this work for their intrinsic correlation to public health affairs. A consolidated discussion comprised the importance of the age of information and the Internet of Things with their existent status in Bangladesh. We have analyzed the component related to COVID-19 in Bangladesh perspective in both figurative and tabular methods. We have statistically analyzed the collected data related to the COVID-19 occurrences in Bangladesh in figurative and expository forms. We analyzed the measures of central tendency and dispersion for the real-time data of COVID-19 components. A more comprehensible analysis of the structure of data of the desired components is exhibited through the Box-Whisker plot with a detailed explanation. The components are the number of tests, infections, deaths, recoveries, quarantines, and isolations. An elaborate discussion on the vaccinations is provided with countywide delineation. Also, a wave-based distribution of the components associated with COVID-19 is displayed. Moreover, some of our findings and suggestions are provided at the end.

It is apparent from the statistical analysis that the COVID-19 component data do not obey the characteristics of a normal distribution and have moderate scatterings. The data's quartiles are not evenly distributed, and their positive skewness has a long right tail that is an indication of initial dominance of the COVID-19 components and the gradual decrease with some irregularities. We have observed that initially, the numbers of infections and deaths were inferior in comparison to the global situation but these increased alarmingly in the first quarter of 2021 and continued for the next half of the year. It happened due to the lack of healthcare sustainability, infirm socio-economic conditions, deficiency of technological advancement, and some troublesome issues caused by illiteracy. The scarcity of basic knowledge about epidemiological diseases and their remedy was another origin of public sluggishness against the combat with COVID-19. Later on, time-worthy moves were taken, and region-wise lockdown and vaccination campaigns triggered substantial preventive outcomes. Also, compatible tactics for quarantines and isolations were pursued and applied throughout the country. The ambience started to change in the fourth quarter of 2021, the number of infections and deaths remarkably declined, whereas the number of recoveries was highly significant which was moderate before. Though in the middle of 2022 another raise of lethal infections were experienced in Bangladesh, it was released quickly, and nowadays, the pandemic ingredients are under control.

## Figures and Tables

**Figure 1:** Statistical analysis of the COVID-19 components.

**Figure 2:** Box-Whisker plot of *Z*-scores.

**Figure 3:** Number of tests.

**Figure 4:** Division-wise number of tests.

**Figure 5:** Number of infections.

**Figure 6:** Division-wise number of infections.

**Figure 7:** Number of deaths.

**Figure 8:** Number of recoveries.

**Figure 9:** Number of quarantines.

**Figure 10:** Number of isolations.

**Figure 11:** Number of vaccinations.

**Figure 12:** Dose-wise number of vaccinations.

**Figure 13:** Type-wise number of vaccinations: (a) First dose. (b) Second dose. (c) Third dose.

**Figure 14:** Division-wise number of vaccinations.

**Figure 15:** District-wise number of vaccinations.

**Table 1:** Waves of the COVID-19 in Bangladesh (https://en.wikipedia.org/wiki/COVID-19_pandemic_in_Bangladesh).

Waves	Start	End
First	March 2020	May 2020
Second	March 2021	May 2021
Third	May 2021	August 2021
Fourth	June 2022	August 2022

**Table 2:** Lockdown of the COVID-19 in Bangladesh (https://betterwork.org/portfolio/covid-timeline-in-bangladesh).

Lockdown	Start	End
First	March 26, 2020	May 30, 2020
Second	April 05, 2021	April 28, 2021
Third	June 28, 2021	August 10, 2021

**Table 3:** Variants of the COVID-19 detected in Bangladesh (https://en.wikipedia.org/wiki/Variants_of_SARS-CoV-2https://www.who.int/en/activities/tracking-SARS-CoV-2-variantshttps://archive.dhakatribune.com/health/coronavirus/2021/05/17/five-covid-variants-found-in-bangladesh-so-far).

Variant	Origin	Date of detection
Beta	South African variant	November 1, 2020
Alpha	UK variant	December 31, 2020
Eta	Indian variant	March 11, 2021
Gamma	Brazilian variant	April 20, 2021
Delta	Indian variant	April 27, 2021
Lambda	South American variant	August 16, 2021
Omicron	South African variant	December 6, 2021

**Table 4:** Vaccinations of different types of vaccines and doses.

Type	First dose	Second dose	Third dose	Total
AstraZeneca	20743272	19254707	11949390	51947369
Pfizer	22306024	20710925	25690994	68707943
Sinopharm	56364937	53985721	217	110350875
Moderna	3778926	3547557	8481643	15808126
Sinovac	27156813	24583986	3371201	55112000
Janssen	0	456284	1053	457337
Pfizer-PF	1250662	0	0	1250662
Total	131600634	122539180	49494498	303634312

**Table 5:** Type-wise maximum daily vaccinations (with date).

Type	First dose	Second dose	Third dose
AstraZeneca	392864 (23/11/21)	439906 (28/03/22)	835985 (06/06/22)
Pfizer	1191272 (13/01/22)	872357 (15/02/22)	5603599 (19/07/22)
Sinopharm	6462094 (28/09/21)	5071068 (28/10/21)	162 (30/06/22)
Moderna	342946 (07/08/21)	386203 (07/09/21)	842651 (05/06/22)
Sinovac	8027784 (26/02/22)	4720122 (28/03/22)	1714618 (29/09/22)
Janssen	0	93302 (26/02/22)	172 (29/09/22)
Pfizer-PF	86929 (29/08/22)	0	0

**Table 6:** Division-wise vaccination coverage.

Vaccination coverage	First dose	Second dose	Third dose
Maximum	Dhaka (87.6%)	Dhaka (78.6%)	Khukna (37.5.%)
Minimum	Barisal (71.5%)	Barisal (64.8%)	Mymensingh (26.8%)
Average	75.3%	70.8%	31.6%

**Table 7:** District-wise vaccination coverage.

Vaccination coverage	First dose	Second dose	Third dose
Maximum	Gazipur (125.6%)	Gazipur (103.9%)	Chuadanga (53.2%)
Minimum	Jhalokati (63.9%)	Shariatpur (60.1%)	Gaibandha (22.2%)
Average	74.8%	70.6%	32.6%

**Table 8:** Wave-wise components of the COVID-19.

Component	Wave 1	Wave 2	Wave 3	Wave 4
Tested	296168	640345	1705258	305632
Infected	44573	117250	493294	36466
Death	607	2039	8989	164
Recovery	9368	119837	430659	41858
Quarantined	Not found	52489	293042	19229
Isolated	Not found	15252	158908	5173

## Data Availability

The data used in this work can be found at the following link: https://github.com/mu2mahmud/Statistical-data-for-Covid-19-in-Bangladesh.
